The article "Long Term Oral Administration of Oregano Essence Effectively Relieves Polycystic Ovarian Rats through Endocrine and Inflammatory Balance" was published in 2022. Journal: Evid Based Complement Alternat Med.

# Long Term Oral Administration of Oregano Essence Effectively Relieves Polycystic Ovarian Rats through Endocrine and Inflammatory Balance

**DOI:** 10.1155/2022/5303583

**Published:** 2022-09-16

**Authors:** Ali Ghorbani Ranjbary, Jalil Mehrzad, Massoud Talebkhan Garoussi, Javad Zohdi

**Affiliations:** ^1^Department of Microbiology and Immunology, Faculty of Veterinary Medicine, University of Tehran, Tehran, Iran; ^2^Department of Theriogenology, Faculty of Veterinary Medicine, University of Tehran, Tehran, Iran

## Abstract

Polycystic ovarian syndrome (PCOS) is alarmingly rising and sustainable therapy/prevention is needed. Here, we evaluated the therapeutic effects of oregano or *Origanum vulgare* (O. vulgare) essence (OE) on the PCOS rat model system. Vaginal smears monitored the estrous cycle of 40 virgin adult rats, and they received 2 mg estradiol valerate (EV)/0.2 ml corn oil intramuscularly to induce PCOS. At 60 days post-EV injection, all rats were evaluated for follicular development/cysts. The EV-induced PCOS rats were orally administered 250 and 500 mg/kgBW/day of OE for 30 days. OE was also further assessed for its predominant components along with hormonal, histological, and inflammatory-related gene expressions in the ovaries. The main components of the OE were predominantly pulegone (36.3), L-menthone (31.3%), far less piperitone (7.8%), isopiperitone (6.4%), isomenthol (3.6%), humulene epoxide II (2.2%), *α*-pinene (1.7%), and thymol (1.5%). Hormonal, histological, and inflammatory-related gene expression results showed >4-fold and 1.5-fold increase in FSH and progesterone; ∼50%, 85%, 45%, 55%, and 30% decreased in LH, estradiol, estrogen, testosterone, and AMH; and dose-dependently decreased in mRNA expression of IL-6, IL-1*α*, NF-kB, TNF-*α*, and IL-1*β* by 25–65%, 55–75%, 15–40%, 30–55%, and 35–55%, respectively, and thus decreased the severity of PCOS, boosted endocrine balance, restored functional follicles and corpus luteum, and thus ovulation in PCOS rats. Overall, in the disrupted PCOS rats, OE oral treatment effectively relieved estradiol-induced PCOS rats via: (1) its endocrine balancing on GnRH, FSH, and LH and (2) its anti-inflammatory and antioxidant properties on ovary caused by OE's useful compounds like pulegone, thymol, and L-menthone. Though many aspects of the effects remain to be tested, such an underlying mechanistic reproductive regulatory effect observed in OE-administered rats further proves its sensible pharmaceutical applications in reproductive medicine and more specifically, PCOS.

## 1. Background

Ovarian cysts are the most common endocrine disorder affecting women and animals' reproduction [1]. Tissue remodeling processes in the ovaries are important in follicular growth, ovulation, and corpus luteum (CL) regression [2]. As one of the main causes of infertility, polycystic ovary syndrome (PCOS) is a reproductive hormonal/metabolic disorder affecting ∼10% of reproductive-age women [3]. Though spontaneous ovulation and pregnancy occasionally occur in women with PCOS, most PCOS cases suffer from chronic anovulation. Generally, PCOS cases show different symptoms; among the most important symptoms are abnormal and irregular cycles, abnormality in facial hair growth, infertility and subfertility, overweight, increase in androgen (clinical or biochemical), anovulation or oligovulation, and dysfunctions in hypothalamus, pituitary, and ovarian glands (accompany by increased LH and testosterone and decreased FSH and estrogen as the main multifactorial disorders) together with insulin resistance [4, 5].

Alternative treatment of female reproductive disorders using herbal remedies is gaining popularity in human medicine [6]. *Origanum vulgare* (*O. vulgare*) or oregano in traditional medicine is used as a disinfectant, antispasmodic, antiflatulent, antiworm, and is also used for liver and gallbladder discomforts [7]. About ∼25 beneficial compounds (i.e., 26.9% thymol, 40.7% carvacrol, and 7.3% gamma Trypnyn) are available in oregano [8, 9], of which phenols, monoterpene hydrocarbons, and alcohol are predominant. Considering the worldwide increasing infertility and medicinal importance of oregano's various effects on the reproductive system, this study was performed to mechanistically pinpoint the beneficial effect of *O. vulgare* (oregano) essence (OE) on hormonal and molecular changes caused by PCOS syndrome in females Wistar rats as a model system for human.

## 2. Materials and Methods

### 2.1. Animals and Housing Conditions and Location of Herb

After one week of acclimatization, 8-week-old adult female Wistar rats (*n* = 40) were divided into 4 groups of 10 rats, consisting of vehicle control group (negative or non-CPOS control), positive control (EV-induced PCOS, received only EV and suffers from PCOS but does not receive any therapeutic substance), EV-induced PCOS with 250 mg OE/Kg, and EV-induced PCOS with 500 mg OE/Kg (to describe the vaginal smear to detect the estrus cycle phases, etc. *n* = 10, but for the experimentation *n* = 3 from each group). Indeed, the administered dosage was determined accordingly [10]; the mentioned concentrations of OE have no side effects in mammalian cells [10]. They were treated in compliance with the guide to the care and use of experimental animals. The weight ranged 180–200 gm. They were nurtured in the professional animal room for a week to be adapted to the environment. Ethical principles of animal care and rights were observed by the Department of Laboratory Animal Breeding, Faculty of Veterinary Medicine, University of Tehran, as well as the authors (IRTU.1399.10.11). The location of the natural herb, *O. vulgare* or oregano, is shown in Figure 1. To study the relationship between the PCOS and sympathetic innervations, the most commonly used PCOS model is generated by a single injection of EV in prepubertal rats done herein, which results in a polycystic ovary morphology, hormonal imbalance, and irregular estrous cycles.

### 2.2. Preparation of Vaginal Smears

Establishing the estrous cycle was followed using vaginal smears, which were obtained between 08:00 and 12:00. They were then evaluated by light microscopy for the relative proportion of leukocytes, epithelial, and cornified cells found in daily vaginal smear (Figures 1(a)–1(f)), which characteristically changes during different stages of the estrous cycle. The rat estrous cycle (estrus, diestrus 1, metestrus, and proestrus) usually took about 4 days, in both control and OE-treatment groups [11].

### 2.3. Oregano Extract Preparation and Analyses

The herb was purchased from a local herb shop in Shiraz-Iran and identified according to the standard protocol. The leaves were cleaned and powdered using an electric blender and then extracted with 75% alcohol for 72 hours using the macerated method. The oregano powder (150 gm) was poured into a one-liter balloon. After adding distilled water, the balloon was connected to the Clevenger apparatus. The OE was extracted by a hydrodistillation Clevenger apparatus for 3 hours. The ratio of EO to the dry weight of the plant was 5%. The obtained EO was stored in dark conditions for further tests and assays. The gas chromatography (GC) device used was made by Agilent USA, a 5-HP capillary column with a length of 30 cm and an inner diameter of 0.25 mm. The oven temperature program was set from 60 to 250 degrees and the mass range from 50 to 250 z/m was recorded. The temperature of the injection chamber, quadrupole mass analyzer, and ionization chamber were set to 280, 150, and 270°C, respectively [12].

### 2.4. GC-Mass Spectrometry Analysis of OE Compounds

Samples were analyzed through GC using an Agilent HP6890 instrument coupled with an HP 5973 mass spectrometer. The GC was equipped with a split-splitless injector and a factor four TM VF-35 ms 5% phenyl-methylpolysiloxane, 30 m, 0.25 mm, and 0.25 *μ*m film thickness capillary column. GC conditions were as follows, temperature range of 60 to 250°C at 40°C/minute, with a solvent delay of 5 minutes along with the injector at 250°C. The inert gas was helium at a flow of 1.0 mL/minute, and the injected volume in splitless mode was 1 *μ*L. The MS conditions were as follows, ionization energy of 70 eV, quadrupole temperature of 100°C, scanning velocity of 1.6 scan/s, and weight range of 40 to 500 amu. The volatile compounds (%) were recorded and qualitative analysis was done based on the percentage area of each peak of the sample compounds. The MS of each compound, which was based on the MS of NIST 98 spectrum library (USA National Institute of Science and Technology Software), was comparatively evaluated as well.

### 2.5. Hormone Treatment Procedures

The experimental rats were included as control and PCOS treatment groups, in which the control rats received an intramuscular (i.m.) injection of 0.2 mlcorn oil and the PCOS rats received an i.m. injection of 0.2 mgestradiol valerate (EV) (Aburaihan Co., Iran) in 0.2 ml of corn oil, to induce PCOS, accordingly [11]. The EV-treated rats were further evaluated 60 days post-injection, during which follicular cells were detected. The PCOS rats were further subdivided into those orally administered: For 30 days, (1) no OE, (2) 250 mg OE/kgBW/day, and (3) 500 mg OE/kgBW/day.

### 2.6. Histopathological Analysis

At the end of the experiment, animals were intraperitoneally (i.p.) injected with a mix of ketamine and xylazin accordingly [13], weighted, and then, 5 mLblood was directly taken from the heart with a syringe (under deep anesthesia and/or euthanasia [14]); afterwards, the abdominal incision was appropriately made. With as much sterile condition as possible (i.e., use of sterile scalpel and forceps and fat removal), the ovaries were isolated and kept in 3% formaldehyde for 2 weeks. Ovaries were imbedded in paraffin; after 5 *μ*m microsections, they were stained with Hematoxylin and Eosin. For this purpose, carefully sliced ovaries were evaluated for follicle count. Then, after every 10 sections, one was selected, and re-counting was done till the last slice was selected for data analysis. 10% of the total sections were randomly counted [15]. The number of primordial, primary, secondary, graph, atretic follicles,and CL were counted byalight microscope with various magnifications. Meannumber of follicles in each group was comparatively specified. The examined healthy or atretic follicles were defined based on their morphology and diameter as follows: (1) primordial follicles (PRIF), where oocyte closely surrounded by one layer of flat granulosa cells,(2) primary follicles (PF), where the growing oocyte is surrounded by one layer of cuboidal granulosa cells, (3) preantral follicles (PAF), where several layers of granulosa cells surround the oocyte with no cavity within, (4) antral follicles (AF), where the oocyte is surrounded by cumulus oophorus cells within the cavity of the antrum, forming, (5)cystic follicles (CF),and(6) CL. Accordingly [16, 17], morphological changes for the evaluation and enumeration of follicles were applied to characterize the follicular atresia and pyknotic nuclei in the granulosa layers; as such, from the basement membrane of oocytes, particularly degeneration of the granulosa layer was apparent in abnormal oocytes.

### 2.7. Measurement of Circulating Gonadotropins and Gonadal Steroids

Blood samples were collected from anesthetized rats' hearts using 5 cc syringes. Blood serum was collected with centrifugation (1000 × *g*, 15 min, 4°C) and stored at −20°Cuntil it was tested. Samples were collected and serum luteinizing hormone (LH), follicular stimulating hormone (FSH), and estradiol levels were determined by the ELISA method. The circulating gonadotropins and gonadal steroids (eg., testosterone (T), progesterone (P), and antimullerian hormone (AMH)) were measured using an ELISA kit (ELISA, DRG, Germany). Testosterone (T), progesterone (P), and anti-mullerian hormone (AMH) were measured using an ELISA kit (ELISA, DRG, Germany).

### 2.8. RNA Extraction and RT-qPCR Assays

In order to determine the expression level of some inflammation-related genes (i.e., NF-kB, TNF-*α*, IL-1*α*, IL-1*β*, and IL-6), the RT-qPCR method was used in the studied rats' ovary. Total RNA from the ovary tissues was extracted using (DENAzist Asia Co., Iran) kit. After analyzing nanodrop and agarose gel electrophoresis, it was converted to cDNA. Indeed, for cDNA synthesis, 1000 ng of total RNA was reverse transcribed into cDNA in a reaction volume of 20 *μ*L using cDNA Synthesis Kit (Yekta Tajhiz Azma (YTA (Cat No: YT4500, Iran)). The expression levels of these inflammatory-related genes (here, NF-*κ*B, TNF-*α*, IL-1*α*, IL1*β*, IL6, and GAPDH, as the reference gene, see below) in ovarian tissues of different groups were assessed by quantitative polymerase chain reaction (qPCR).

After obtaining exon sequences from NCBI (National Center for Biotechnology Information) and Ensembl, the required primers were designed on two exons or as forward or reverse on the junction of two exons by Beacon Designer v8. Then, using Beacon, Oligo, and NCBI, Primer-BLAST was performed and primers were checked for the position and extra bands. Then, after ordering and purchasing the designed primers, they were diluted and used according to the manufacturer's protocol. Details of designed primers are as follows: for NF-*κ*B, F: 5′-TAATGCTTACACGGACTT-3′ and R: 5′-CCCATCCTTATTCTTTATGC-3′; for TNF-*α*, F: 5′-CTCCCTCTCATCAGTTCCAT-3′ and R: 5′-GCTACGGGCTTGTCACTC-3′; for IL-1*α*, F: 5′-TTAGAAGAGACCATCCAA-3′ and R: 5′-TGTATTCTGTCCATATCCA-3′; for IL1*β*, F: 5′-GACCCAAGCACCTTCTTT-3′ and R: 5′-TAGCAGGTCGTCATCATC-3′; for IL-6, F: 5′-ATTGTATGAACAGCGATGAT-3′ and R: 5′-AGAAGACCAGAGCAGATT-3′; and for GAPDH, F: 5′-ATGTTCCAATATGATTCCA-3′ and R: 5′-GATTTCCATTGATGACAAG-3′. qPCR was performed using SYBR Green qPCR Master Mix (amplicon). The qPCR conditions for all genes were carried out (in triplicates) with a cycling program including holding for 10 min at 95°C, followed by 40 cycles of 95°C for 10 sec, annealing at 60°C for 20 sec, and 72°C for 20 sec. Melting curve analysis and agarose gel electrophoresis were also performed to ascertain the specificity of the reactions or the absence of nonspecific PCR products (data not shown). By using GenEx 6 software, data were analyzed according to the comparative Ct (2^−ΔΔCt^) method as fold change relative to the expression level of control samples.

### 2.9. Statistical Analysis

The data were expressed in SI units and analyzed by repeated measurements ANOVA, Duncan, Spearman, and *t* test using GraphPad Prism 8 software. All the experiments were performed in duplicate with the results of three independent experiments. The values were then expressed as mean and standard error of mean (SEM), and *P* < 0.05 was seen as statistically significant.

## 3. Results

Figure 1(a) shows the distribution of oregano in the region (Iran). Twenty-one chemical compounds were identified. Among these, 5 compounds make up the most predominant oregano chemicals are pulegone (36.3%), L-menthone (31.3.53%), piperitone (7.8%), isomenthol (3.6%), and thymol (1.51%) were present in the respective decreasing order (Figure 1(b)).

### 3.1. Oregano Essence Boosts Normal Ovarian Morphology in PCOS

Each phase of the estrous cycle was identified by the presence of three types of cells: numerous nucleated epithelial cells in the proestrus phase; nonnucleated cornified cells in the estrous phase; nucleated epithelial cells, nonnucleated cornified cells, and leukocytes in metestrus phase, and plenty of leukocytes in diestrus phase. Figures 2(a)–2(f) of rat show vaginal smears from the non-PCOS control group in the proestrus (Figure 2), estrus (Figure 2(b)), metestrus (Figure 2(a)), and diestrus (Figure 2(d)) phases; from the EV-induced PCOS group, the vaginal smears predominantly exhibited leukocytes, the main cells observed during the diestrus stage (Figure 2(e)), and the EV-induced PCOS + 500 mg/kg oregano group exhibited epithelial keratinocytes, the main cell type observed during the estrus stage (Figure 2(f)).

In the ovaries of rats treated with OE treatment, large cystic follicles with a narrow granulosa layer of one or two cell layers and a small number of small follicles characteristic of PCOS were observed (Figure 2(h)); no CL was observed in this group. Unlike the OE-treated rats, in the control group, the ovaries had no cysts and were full of CL, indicating normal ovulation in this group. Also, the number of small follicles was much higher. Therefore, based on our observations, treatment with OE after 60 days led to the normal formation of cysts and ovulation in the OE-treated group. Also, morphological examinations of post-OE treated PCOS showed a number of CL, indicating the beginning of ovulation in the OE-treated groups. A marked increase in small follicles was observed between the OE-treated PCOS and PCOS rats. After treatment of PCOS ovaries with OE, morphological examinations showed that the number and size of cysts decreased, CL appeared, and the number of small follicles in OE-treated PCOS groups was higher than in the control group (Figures 2(g)–2(j)). In PCOS ovaries treated with 250 mg OE/kg, various follicles including antral and corpus luteum (small number) were observed (Figure 2(i)). Cross-sectional examination of the ovarian of the PCOS group treated with 500 mg OE/kg antral follicles, parenteral and grown follicles were observed (Figure 2(j)).

### 3.2. Effects of Oregano Essence on Oocytes in PCOS Rat

The number of immature oocytes that reached metaphase II in the PCOS group was significantly lower than in the control group. However, in the groups receiving 250 and 500 mg/kg of OE, the number of dividing oocytes increased compared to PCOS (see Figure 3). The number of primary follicles (15.56 ± 0.63) and antral follicles (7.35 ± 1.2) and CL (9.45 ± 1.65) were normal (Table 1). However, in PCOS group, numbers of primary follicles, antral follicles, cystic follicles, and CL were 5.36 ± 1.2, 2.36 ± 1.1, 6.87 ± 1.25, and 1.9 ± 1.2, respectively. Ovarian treatment by oregano was additionally confirmed by the count of follicles and CL in 250 mg/kg and 500 mg/kg groups. In 500 mg/kg group numbers of primary follicles, antral follicles, cystic follicles, and CL were 14.96 ± 1.2, 6.96 ± 1.36, 0, and 9.85 ± 1.97, respectively (Table 1).

### 3.3. Oregano Essence Improved Serum Sex Steroids in PCOS Rat

Compared to EV-induced PCOS group, serum levels of LH, estradiol, estrogen, testosterone, and AMH in the 500 mg/kg of OE significantly decreased by ∼50%, 85%, 45%, 55%, and 30%, respectively (Figure 4). However, serum levels of progesterone and FSH increased in groups of 250 mg OE/kg (∼1.3-fold and 1.7-fold, *P*=0.014 and *P* < 0.0001) and 500 OE·mg/kg (∼4.1-fold and 5-fold, *P* < 0.0001), respectively (see Figure 4).

### 3.4. Oregano Essence Alleviates the Inflammatory Microenvironment in PCOS

Inflammatory-related gene expression of the ovarian tissues results showed a dose-dependent (250–500 mgOE/kg) decrease in the mRNA expression of IL-6, IL-1*α*, NF-kB, TNF-*α*, and IL-1*β* by 25–65%, 55–75%, 15–40%, 30–55%, and 35–55%, respectively, compared to EV-induced PCOS group (see Figure 5). Expression of these genes in the ovarian tissues of the experimental rats was significantly higher (*P* < 0.0001) in EV-induced PCOS than the negative (healthy) control group (Figure 5). Indeed, in rats with PCOS receiving OE, inflammatory markers remarkably downregulated in a dose-dependent manner compared to those of non-OE treated PCOS rats (*P* < 0.0001, Figure 5).

## 4. Discussion

In the present study, the effect of oregano essence, which has antioxidant compounds with potential anti-inflammatory properties, on the improvement of PCOS induced by EV was investigated. The analytical results showed that OE contains antioxidant compounds such as pulegone and thymol. Also, PCOS treatment with OE reduced serum levels of LH, AMH, estradiol, and testosterone. Additionally, the application of hot aqueous *O. vulgare* enhances the female murine reproductive performance [18]. In the present study, we used EV for the induction of PCOS in adult female rats. Following induction of PCOS, estradiol and testosterone significantly increased, while the level of progesterone significantly decreased in EV-induced PCOS rats with almost little change in seral dehydroepiandrosterone (DHEA). Such a finding with EV-induced PCOS is in line with the findings by other researchers [19, 20].

With hugely complexed etiology and worldwide affecting ∼8% of women, PCOS is the most common cause of female infertility. The OE-administered induction of hormonal balance, histological normality, anti-inflammatory microenvironment of the ovary and decreased severity of PCOS, boosted endocrine balance, restored functional follicles and CL, and thus ovulation in PCOS rats, strongly leading us to apply this medicinal plant for pharmaceutical applications.

Our qPCR results showed that the pro-inflammatory genes expression increased in ovarian tissues of EV-induced PCOS groups compared to the healthy non-PCOS control group and different doses of OE-treated PCOS group. In all OE-treated PCOS rats, it was obvious that OE alleviated PCOS by suppressing inflammation through downregulating the expression levels of inflammation-related genes, including TNF-kB, TNF-*α*, IL-1*α*, IL-1*β*, and IL-6. The finding here is in line with the other findings, showing reduced inflammation and inflammatory-related genes in LPS-affected THP-1 cells [21]. Indeed, inflammatory-related gene downregulation observed herein strongly confirms the decreased severity of PCOS caused partially by inflammation; though many aspects of the effects of inflammatory molecules remain to be tested; nonetheless, such an underlying mechanistic reproductive regulatory effect observed in OE-administered PCOS rats further proves the OE's sensible pharmaceutical applications in reproductive medicine.

The multifactorial etiology of follicular PCOS is obvious (i.e., pathological (inflammation and infections), physiological, nutritional, metabolic, obesity, and diabetes etcetera) in human, monkey, rodents, farm animals; in all forms of PCOS, the disruption of hypothalamic-pituitary-gonadal (HPG) axis along with hyperandrogenism, anovulation, presence of multiple ovarian cysts, irregularities in the menstrual cycle, variable levels of gonadotropins and particularly increased blood levels of estradiol occur. Several experimental models have been proposed to induce PCOS in neonatal, prepubertal, or adult rats, depending on the phenotypic, genetic, environmental, and physiological characteristics such as steroidal and nonsteroidal drugs (dehydroepiandrosterone, dihydrotestosterone, letrozole, and estradiol valerate (EV)-administration) and manipulations (genetically modified rat models as well as models developed with exposure to constant light or stress) that are to be investigated. What triggers the PCOS and what exact time of the estrus cycle the PCOS occurs in rat are hugely complex and somewhat unclear, but in nature, the main starting point of PCOS is puberty and sexual maturation; we did not evaluate and address the exact time of PCOS occurrence; nonetheless, the quantification of progesterone levels before the induction of PCOS with EV is valuable to figure out the exact time of PCOS occurrence. It is worth mentioning that all healthy experimental rats were sexually mature. It is therefore necessary to measure progesterone on the daily basis to know the exact phase of the estrus cycle. To our experience in farm animals like cattle, the PCOS normally occurs after parturition, which always accompanied by mild uterus infection/inflammation, in which we normally use intrauterine antibiotic therapy to relieves PCOS in cattle. As such, mild inflammation would be one of the underlying causes of PCOS and anti-inflammatory approach of the reproductive system would surely relieve the PCOS.

Experimental PCOS in rodents resembles some aspects of the human PCOS syndrome; in one example, long-acting EV changes serum levels of gonadotropin-releasing hormones (GnRH) and induces the appearance of follicular cysts. Neuroendocrinologically, the neuronal component responsible for the induction of the LH surge is located in the preoptic area (POA) in female rats [22]. Indeed, GnRH neurons in the POA express the immediate early gene, c-Fos, at the time of the LH surge, suggesting that such POA-associated GnRH neurons are responsible for the GnRH surge [23]. Mechanistically,LH surge (i.e., the GnRH surge) ishugely linked to the neural parts of the GnRH generator. This neural-related regulation of LH surge, in turn, also links to gamma amino butyric acid (GABAergic) regulation machinery[24]. Accordingly[25], a decrease in the inhibitory tone of GABA on GnRH neurons causes LH surge[26].That is whymorning i.v. infusion of bicuculline, a GABAA receptor antagonist, during the proestrus phase remarkably induces a premature surge-like secretion of LH. The significant proportion of beneficiary molecules like phenols, monotropone hydrocarbons like P-simine, Y-tripine, linalul, x-tronpine, and thujan 4–01 [27] and other antioxidant compounds like thymul, cavacrol, linalool, camphan, and toylen [28] in OE might have caused such beneficial effects.

Results of the present study also showed that OE treatment increases serum levels of progesterone and FSH in EV-induced PCOS rats. This can be helpful for PCOS subjects/human/mice/rat duemainly to the point that progesterone levels decreased in PCOS mice [29] as also observed herein. Indeed, ovarian tissue changes in the PCOS group in the present study were consistent with others [30–32], indicating the successful induction of PCOS with EV and defects in the development of follicular clusters in adult rats compared to the non-PCOS control group. Also, it seems that angiogenesis is likely due to increased expression of vascular endothelial growth factor and isoenzyme 2 cyclooxygenase in the stroma; this was also confirmed by observing a follicular increase in the sheath layer and androgen production or progression of steroidogenesis with thickening of this layer [11, 30].

Since androgens are considered the main source of PCOS, and androgenization of animals is the most frequently used approach to induce PCOS, of which characteristics include anovulation, cyst-like follicles, elevated LH levels, increased adiposity, and insulin insensitivity (31). Most commonly used androgens in mouse models of PCOS are testosterone, DHEA, and dihydrotestosterone (DHT). However, estrogen treatment has also been applied as we did herein. The timing of androgen exposure varies widely, starting as early as prenatal exposure. Further, neonatal, prepubertal, and adult androgenization of mice has been applied. Since clinical symptoms of PCOS often start during puberty [32], treatment of mice before adulthood will likely be more closely resembled PCOS in human. Indeed, androgens-based GnRH pulsatility was observed in neonatally-induced model of PCOS. In PCOS, GnRH pulse frequency is increased; this implies that androgens may reprogram the steroidal feedback on GnRH neurons, resulting in GnRH neuron hyperactivity (31, 32). Therefore, the increased GnRH pulsatility makes it an interesting model to study the reprogramming effect of androgens on the HPG axis. The impact of OE on such interestingly complex events of HPG axis and thus PCOS remains to be further examined.

Considering the inhibitory effects of flavonoids, thymol, and menthol (as important compounds in the OE of this plant family) on cyclooxygenase enzymes, it is acceptable that the compounds in OE improve the ovarian tissue symptoms in PCOS rats by inhibiting follicular sheath cell proliferation. Nonetheless, it is worth assessing the fluctuations on the isoenzyme 2 cyclooxygenase in OE-(un) treated PCOS individuals.

About the safety concerns of the oregano, it is indeed widely consumed in Iran and other Asian countries as a medicinal plant in the form of tea and tablets for wide range of (non)infectious diseases (its antibacterial and anticancer effects). It also has therapeutic properties. In our previous works, the MTT of this medicinal plant was tested *in vitro* and with high safety range (7). Indeed, oregano would have caused such an observed relieving effect on the POC rats. Therefore, the effects of observed OE in rats can be attributed to the direct activation of the central benzodiazepine and thus opens new windows to understanding molecular mechanisms that might underpin the oregano's components (Figure 6) for reproduction performance. In the disrupted PCOS rats, OE oral treatment effectively relieved estradiol-induced PCOS rats via: (1) its endocrine balancing on GnRH, FSH, and LH, (2) its antioxidant properties ontheovary caused by OE's useful compounds like pulegone, thymol, and L-menthone, and (3) its huge anti-inflammatory properties. Our work here is novel and it is worth to comparatively assess the effect of most suitable doses of OE on the reproduction performance in female reproductive system of the economically important farm animals and humans. To yield more valuable impacts of the administration of the OE for treatment of PCOS, the dosage of 500 mg OE/Kg would be suitable. In short, oregano and its compounds can be useful regulators of ovaries that boost efficient oogenesis, further proving its sensible application in reproductive medicine. Though many aspects of the effects remain to be tested, such an underlying mechanistic reproductive regulatory effect observed in OE-administered rats further proves its sensible pharmaceutical applications in reproductive medicine.

## 5. Conclusions

In conclusion, the finding herein highlighted the beneficial values of the oregano for alleviating PCOS, though somewhat a dose-dependent manner; it can be concluded that the 500 mg OE/kg can be effective in improving of the PCOS symptoms, leading to the orientation of the PCOS ovaries towards the normal ones. The improving effects of OE on PCOS ovarian rats are mainly impacted through HPG axis, functional hormones, antioxidant, and anti-inflammatory properties. The antioxidant compounds in OE should also be noticeable as points of its relieving impacts on PCOS. Since the incidence of PCOS is increasing both in humans and farm-and-companion animals, it is likely that pharmaceutical implications of oregano can be a good drug of choice for endocrine balance and ovarian dys/malfunctions.

## Figures and Tables

**Figure 1:** Location and the used plant oregano (*Origanum vulgare*) in the study. (a) Fresh and dried plants form the nature (plant gathering location in Iran), (b) GC/MS analyses of oregano essence (OE), which was predominantly composed of viridulum chromatogram. Thymol, pulegone, and L-menthone.

**Figure 2:** (a–f): Dried plants in shade area; drying plants in shade. Effect of oregano in the estrous cycle in rats with polycystic ovarian syndrome (PCOS). The representative picture of rat vaginal smears from the non-PCOS control group in proestrus (a × 200), estrus (b × 200), metestrus (c × 200), diestrus (d × 200), from the estradiol valerate (EV)-induced PCOS group predominantly exhibited leukocytes, the main cells observed during the diestrus stage (e × 200), the EV-induced PCOS + 500 mg/kg oregano group exhibited epithelial keratinocytes, the main cell type observed during the estrus stage (f × 200). NE: nuclear epithelial cell, EK: epithelial keratinocyte, L leukocyte. Histological analysis of ovaries reveals oregano's extract boosts ovarian performance in rats; decrease early preantral but increase compact follicles in PCOS rats (g), normal size and structure of follicles in control rats (h), with increased granulosa cells but decrease compact follicles PCOS + 250 mg/kg oregano (*Origanum vulgare*) (i) and EV-induced PCOS + 500 mg/kg oregano (j) groups with normal size (25 *μ*m) of compact follicles; stained with hematoxylin and eosin, ×400; yellow arrows show the early preantral follicles.

**Figure 3:** Oregano essence (OE) oral treatment effectively relieves polycystic ovarian rat via its endocrine balancing and antioxidant properties. Impact of OE on oocytes structural changes, rat oocytes with ×100 magnification by a light microscope. Comparisons of ovarian follicles of four groups. (1) Nonpolycysticovarian syndrome (PCOS) control, Denuded healthy oocytes (DO), (2) estradiol valerate (EV)-induced PCOS, (3) EV-induced PCOS + 250 mg/Kg oregano treatment, and (4) EV-induced PCOS + 500 mg/Kg oral OE treatment groups.

**Figure 4:** Oregano essence (OE) oral treatment of pubertal and adult female mice for 30 days resulted in elevated serum testosterone in comparison with the nonpolycysticovarian syndrome (PCOS) control group in EV-induced PCOS, EV-induced PCOS + 250 mg/Kg, and EV-induced PCOS + 500 mg/Kg, respectively. Oregano oral treatment of adult female mice resulted in decreasing Progesterone Estrogen levels. However, the level of antimullerian hormone (AMH) decreased. Data are mean ± SD of 3 independent experiments with related *P* values.

**Figure 5:** Some inflammatory-related gene overexpression in ovarian tissues of estradiol valerate (EV)-induced polycystic ovarian syndrome (PCOS) rats and improving impact of long term oral administration of oregano essence (OE). OE reduces mRNA expression of NF-kB, TNF-*α*, IL-1*α*, IL-1*β*, and IL-6 in ovarian tissues of estradiol-induced polycystic ovaries rats. Data are mean ± SD of 3 independent experiments. ^*∗∗∗*^*P* < 0.0001 compared with the PCOS group.

**Figure 6:** Representative scheme of the major elements of the neuroendocrine, hypothalamic-pituitary-gonadal (HPG) axis, controlling ovary functions. Hypothalamic GnRH neurons release GnRH to the hypophysial portal blood system and dictates the pulsatile secretion of gonadotropins, LH and FSH that stimulate the maturation and regulate ovaries functions, and thus ovulation led by FSH. LH hormone ensures egg release to the uterus and thus secretion of progesterone by CL. (Adapted from [21–23]). In polycystic ovarian (PCOS) mammals the reproductive regulation is remarkably disrupted with higher levels of GnRH, FSH and LH, and oral administration of oregano essence (OE) effectively relieves estradiol-induced PCOS rat via: (1) its endocrine balancing on GnRH, FSH and LH and (2) its antioxidant and anti-inflammatory properties on ovary caused by OE's useful compounds like pulegone, thymol, and L-menthone. Such a reproductive regulatory effects could translate in OE-administered mammals *in vivo*, of which underlying mechanisms remains to be tested.

**Table 1:** The count of follicles and CL in 4 studied groups.

Experimental group	Primary follicles	Preantral follicles	Antral follicles	Cystic follicles	CL
Non-PCOS control	15.56 ± 0.63^a^	8.12 ± 1.53^a^	7.35 ± 1.2^a^	0^a^	9.45 ± 1.65^a^
EV-induced PCOS	5.36 ± 1.2^b^	2.12 ± 0.36^b^	2.36 ± 1.1^b^	6.87 ± 1.25^b^	1.9 ± 1.2^b^
EV-induced PCO + 250 mg/kg oregano	11.36 ± 0.92^a^	6.34 ± 0.74^a^	3.63 ± 1.53^a^	1.96 ± 1.1^a^	6.12 ± 1.52^a^
EV-induced PCO + 500 mg/kg oregano	14.96 ± 1.2^a^	8.64 ± 1.45^a^	6.96 ± 1.36^a^	0^a^	9.85 ± 1.97^a^

are presented as mean ± SD of 3 independent experiments, *t*-test. Different letters show a notable difference with other groups (*P* < 0.05). Polycystic ovarian syndrome (PCOS), estradiol valerate (EV), corpus luteum (CL).

## Data Availability

The data used to support the findings of this study are available upon request.
